This article has been retracted.

# Image Analysis Application of Motherwort Total Alkaloid Injection in the Treatment of Postabortion Hemorrhage

**DOI:** 10.1155/2022/8725030

**Published:** 2022-03-24

**Authors:** Wenjing Wang

**Affiliations:** Shaanxi University of Chinese Medicine, Xianyang, Shaanxi 712046, China

## Abstract

In order to reduce the possibility of postabortion hemorrhage leading to maternal death, the author studied the image analysis of postpartum hemorrhage based on *Leonurus* total alkaloid injection, combining research results, in order to explore the curative effect of *Leonurus* injection in treating postpartum hemorrhage. After treatment, the time and volume of vaginal bleeding were significantly lower than those in the control group (*P* < 0.05); it is suggested that the combination of oxytocin and motherwort can effectively reduce the time and volume of vaginal bleeding after medical abortion, conducive to postoperative recovery. The results show that motherwort injection can effectively reduce the amount of bleeding and reduce the risk of postpartum hemorrhage; in addition, adverse reactions have been reduced, and an image analysis consensus has been formed, which is worthy of promotion.

## 1. Introduction

Motherwort is the above-ground part of the motherwort, a plant of the Lamiaceae; its taste is bitter, pungent, and slightly cold in nature. It is returned to the liver, pericardium, and bladder meridian; it has the effects of promoting blood circulation, regulating menstruation, promoting hydration, and reducing swelling, clearing away heat and detoxification. Often used to treat irregular menstruation, dysmenorrhea, amenorrhea, endless lochia, edema, oliguria, carbuncle swelling, and poison. Zhang Jingyue's “Materia Medica” discusses “blood qi element deficiency and cold, and those who have slipped and are not solid are not suitable;” clinical adverse drug reactions (ADR) reported that long-term large-scale use of motherwort caused kidney damage and so on [1]. Motherwort alkaloid (AFL) is the main chemical and medicinal substance; preliminary studies have proved that the total alkaloid content has a certain correlation with toxicity; however, there are few studies on the toxicity of AFL, the characteristics of its toxic effects in the body, the spectrum of toxic effects, pathways of toxic effects, biological mechanisms, and in vivo processes that can identify the basis of substances; studies on the relationship between blood drug concentration and toxic and side effects are still blank, and this greatly restricts the safe use of motherwort [2]. The high incidence of postpartum hemorrhage is an important cause of maternal death in my country; uterine weakness is the primary factor causing postpartum hemorrhage; the application of fast, safe, and effective uterine contraction agents is still the fundamental method for obstetricians to deal with uterine weakness; the main causes of postpartum death are shown in Figure 1. Motherwort injection is a modern pure Chinese medicine preparation derived from “good medicine for economics and production” motherwort; it has synergistic and complementary effects with oxytocin and other oxytocins; it can promote the contraction of smooth muscle of the whole uterus, without receptor saturation. The main effective chemical components of its contraction effect are motherwort alkaloids and so on [3]. Ultrasound image examination: scanning the pelvic cavity from multiple angles focus on observing the shape and size of the uterus, whether there are abnormal echoes in the myometrium and uterine cavity, and whether there are other abnormalities in the double appendage area and the pelvic cavity. When an abnormal echo is found in the uterine cavity or muscle layer, record its location and scope in detail and use color and spectral Doppler to detect its blood flow; when the arterial blood flow spectrum is collected, with its resistance index (RI), pulse index (PI), and peak systolic velocity (PSV), when sampling multiple times, the final data are the maximum value of PSV [4]. Domestic perinatal medicine, clinical pharmacy, evidence-based medicine, and experts from various clinical related disciplines jointly drafted and formulated the “Consensus on the Application of Motherwort Injection in the Prevention and Treatment of Postpartum Hemorrhage,” for reference to physicians and pharmacists in clinical works to further standardize the clinical application of *Leonurus* injection, in order to achieve more ideal results and benefit more patients [5].

## 2. Literature Review

Huang Qingfang and others used the BL-420E + biological signal acquisition and processing system, studied the effects of motherwort fat-soluble alkaloids and water-soluble alkaloids on the tension of isolated uterine smooth muscle in mice, and the result shows that motherwort fat-soluble alkaloids have a certain inhibitory effect on isoproterenol-induced uterine contractions in vitro (*P* < 0.05). Motherwort water-soluble alkaloids on propranolol, diphenhydramine, and nifedipine caused a certain excitatory effect on isolated uterine relaxation (*P* < 0.01) [6]. Among them, the inhibitory effect of the fat-soluble alkaloids of motherwort on the uterus may be related to *β*-receptors. The excitatory effect of the water-soluble alkaloids and total flavonoids of *Leonurus* on the uterus may be related to H1 receptor and *β* receptor Ca^2+^-ATPase [7]. It is also reported that with leonurusine hydrochloride 0.03, 0.06, and 0.09 mg mL^−1^ and stachydrine hydrochloride 0.12 and 0.18 mg mL^−1^, the isolated rat uterine spasm caused by oxytocin is inhibited and synergistically enhanced [8]. Motherwort injection mainly contains the total alkaloids of motherwort; the study found that motherwort injection extract can increase the vitality and contraction tension of the isolated uterus of aborted rats (*P* < 0.01); it is the main active part of promoting abortion uterine contraction and inhibiting abortion uterine contraction, and it is the water-soluble alkaloid site of motherwort, which has the effect of increasing the minimum tension of aborted uterine contraction (*P* < 0.05); it is the main material basis for motherwort injection to exert uterine contraction [9]. Liu et al. conducted an ultrasound image scanning study on the active part of the uterine contraction of *Leonurus* injection and found that the active parts of the excitement uterus are B1 (mainly hydrazine), B2 (mainly hydrazine, fenugreek), and B4 (mainly contains fenugreek, choline, and total amino acids), and the part of the diastolic uterus is B3 (mainly containing fenugreek and choline). The study found that no matter if motherwort injection is used alone or combined with oxytocin, both can effectively prevent and treat postpartum hemorrhage during normal delivery and uterine delivery [10]. Yu Changli and others used motherwort injection combined with oxytocin after delivery of the fetus's anterior shoulder, immediately intramuscular injection into the hip to prevent and treat postpartum hemorrhage after delivery; the results show that the combination of drugs is significantly better than the single use because the onset of oxytocin is fast, but its half-life is short (3-4 min), and the maintenance time is short, and motherwort injection has a slower onset, but has a long-lasting uterine contraction and hemostasis effect; the combined effect is complementary, the hemostatic effect is obvious, and it has the function of promoting uterine involution [11]. Zhou Yuanyang and others used motherwort injection (1 and 2 mL) to inject intramuscular injection of cesarean section to prevent and treat postpartum hemorrhage; the results show that both doses of injection can promote uterine contraction, significantly reduce postpartum hemorrhage, and the 2 mL group is better than the 1 mL group in reducing postpartum hemorrhage; its hemostatic mechanism may be related to the increase of estrogen levels [12]. Li et al. used motherwort injection combined with oxytocin, and compared the ultrasound image scanning effect of oxytocin alone in the prevention and treatment of postpartum hemorrhage of cesarean section; it was found that the bleeding volume of the combined medication group was less than that of the oxytocin group at 0–2, 2–24 h after surgery, and reduce the occurrence of adverse reactions, and analyze the causes of contractions as shown in Figure 2. Lishun et al. used different extracts of motherwort to study the effect of rabbit blood viscosity; it was found that the total alkaloids of motherwort can significantly reduce the blood viscosity of rabbits, dilate tiny blood vessels, and improve microcirculation [13]. Ding Boping used subcutaneous injection of high-dose epinephrine and ice-cold bath to make a blood stasis model in rats and observe the effects of leonurusine on blood rheology and other indicators in the blood stasis model of rats. The results show that leonurusine (6.0, 3.0, and 1.5 mg kg^−1^) in each dose group can significantly reduce blood viscosity and improve the deformability of red blood cells [14]. The effect of leonurusine on hemorheology may be related to the dilation of blood vessels and the reduction of fibrinogen content. Motherwort injection is a colorless liquid of 20 mg hydrazine per 1 mL obtained by water extraction and alcohol precipitation of motherwort, advantageous formulation developed for motherwort, and it is widely used clinically to prevent and treat postpartum hemorrhage and promote postpartum uterine involution [15]. Qin Xianfen reported that the half-life of oxytocin is 1–6 minutes, motherwort injection is about 6 hours, and the combination of the two has a synergistic effect; when the effect of oxytocin diminishes, motherwort injection can still promote uterine contractions and enhance the hemostatic effect; it can effectively avoid the slow onset of motherwort [16]. Another report shows that oxytocin combined with motherwort injection can prolong the contraction time, effectively reduce bleeding, and promote uterine involution [17].

On the basis of the current research, this study, based on the above preliminary research results, suggests that motherwort injection can stimulate the uterus in vitro, and its effective components are alkaloid parts, which is also an important basis for the author to choose the total alkaloid of motherwort injection for related research.

## 3. Research Methods

Prevention and treatment of postpartum hemorrhage is an important means to reduce maternal mortality; the definition of postpartum hemorrhage is not exactly the same in different countries, regions, and different organizations. In our country, after scanning the ultrasound image, it was found that postpartum hemorrhage refers to the bleeding volume of vaginal delivery ≥500 mL within 24 hours after the fetus is delivered, or cesarean section ≥1000 mL, it is the most common and serious complication after delivery [18]. According to the time of occurrence, postpartum hemorrhage can be divided into primary (early stage, within 24 h of delivery) and secondary (late stage, within 24 h of delivery, within 24 h) postpartum hemorrhage [19]. Postpartum hemorrhage is the top four causes of maternal death; it is reported that 34% of global maternal deaths in 2019 were caused by hemorrhage. In 2019, postmanufacturing bleeding accounted for 21.1% of maternal deaths; it has always been the leading cause of maternal death in our country [20]. With the implementation of China's two-child policy, according to the National Women's and Children's Health Report, in 2021, the proportion of pregnant women ≥35 years old nationwide will rise to an unprecedented 17.13%, the proportion of maternal women is as high as 84.07%, and among them, 44.69% of elderly pregnant women are with a history of cesarean section as a high-risk group of postpartum hemorrhage; this undoubtedly brings greater challenges to the prevention and treatment of postpartum hemorrhage. Therefore, effective prevention and treatment of postpartum hemorrhage is the current focus of obstetric clinical practice [21]. The most important thing now is motherwort injection and oxytocin. The difference between the two is given in Table 1.

### 3.1. Objects and Methods

The study subjects and groups were selected from January 1, 2021, to August 31, 2021, with 120 cases of missed abortion patients admitted to the hospital. The patients were randomly divided into the observation group and control group using a random number table, 60 cases in each group. This study complies with medical ethics requirements and has been reviewed and approved by the hospital ethics committee.

### 3.2. Diagnostic Criteria

Diagnostic criteria are referred and obtained from “Obstetrics and Gynecology” published by People's Medical Publishing House in 2015: missed abortion refers to the death of an intrauterine embryo or fetus that is not discharged in time [22].

Inclusion criteria: meet the diagnostic criteria for missed abortion; after abortion with mifepristone combined with misoprostol, uterine evacuation was performed; be informed of this research and sign an informed consent form; vaginal bleeding is less than normal menstrual volume; complete clinical data; and patients who have good compliance and cooperate with research investigations.

Exclusion criteria: those who do not meet the diagnostic criteria for missed abortion; patients suffering from serious genetic, physical, or mental illness; patients with abnormal development of reproductive organs (such as mediastinal uterus); patients with massive vaginal bleeding; ultrasound image scanning does not cooperate with the researcher; patients with severe infectious diseases; patients with severe cardiovascular disease and liver and kidney dysfunction; those who are allergic to the drugs in this study; and incomplete clinical data, which affect the efficacy and safety judgment.

The specific bleeding rate in these 120 cases is shown in Figure 3:

### 3.3. Treatment Methods

#### 3.3.1. The Control Group Was Given Capsule Treatment

Usage: from the first day after Qing Dynasty surgery, fresh motherwort capsules (produced by Zhejiang Dade Pharmaceutical Group Co., Ltd., approval number: National Medicine Standard Z20080052) were taken orally, twice a day, 1.6 g each time for 7 days, and then ultrasound image scan.

#### 3.3.2. The Treatment Group Was Treated with *Leonurus* Injection

Prescription composition: Angelica 10 g, Chuanxiong 10 g, Peach kernel 10 g, Paojiang 6 g, Roasted licorice 6 g, and motherwort 20 g, 1 dose a day, decoction 200 mL (decoction uniformly by the preparation room of our hospital, divided into 2 bags, 100 mL each), divide 2 times, 100 mL each time, for 7 days, and then perform ultrasound image scanning.

Observation index: observe the vaginal bleeding time of the two groups of patients (the duration from the time of vaginal bleeding to the time of cleansing) and the situation of intrauterine hemorrhage in the first week after uterine purgation (the manifestation of intrauterine hemorrhage: intrauterine cavity exploration and width ≥1.5 cm, edge echo enhancement, irregular, and scattered dark areas with strong light spots); among them, the image display of the uterine cavity hemorrhage is uniformly tested by the color Doppler ultrasound room of the hospital [23].

### 3.4. Statistical Methods

Use SPSS 21.0 statistical software for statistical analysis of data. The measurement data are expressed by mean ± standard deviation (−*x* ± *s*). Count data are expressed by rate, and comparison between groups is by the *χ*^2^ test; the rank sum test was used to compare the rank data between groups [24]. The difference was statistically significant with *P* < 0.05.

### 3.5. Safety Issues of Motherwort Injection

Theoretically speaking, motherwort injection may have slight adverse reactions, but the incidence is low. The results of a large sample safety monitoring study involving more than 10,000 cases of 42 hospitals across the country showed that the adverse reaction rate of *Leonurus* injection is 7.9/10000, which is rare [25]. In this study, there were no adverse reactions in the patients who used motherwort injection; it is estimated to be related to the clear material basis and high purity of motherwort injection, but pay attention to observation during clinical use; once symptoms such as fever, chills, rash, gastrointestinal reactions, and arrhythmia occur, it is recommended to stop using [26].

## 4. Results

Comparison of the baseline data of the two groups of patients is as follows. Among the 60 patients in the observation group, age is (32.04 ± 0.17) years old, bodyweight is (55.92 ± 0.20) kg, height is (161.62 ± 0.10) cm, pregnancy times are (1.31 ± 0.02) times, and the parity is (1.04 ± 0.01) times. Among the 60 patients in the control group, the age was (32.00 ± 0.24) years, bodyweight is (55.95 ± 0.20) kg, height is (161.60 ± 0.11) cm, pregnancy times were (1.34 ± 0.02) times, and parity times were (1.03 ± 0.01) times. In comparison of baseline data of the two groups of patients, such as age, bodyweight, height, pregnancy, and parity, the differences were not statistically significant (*P* > 0.05), and they were comparable. The comparison of motherwort injection before and after use is shown in Figure 4.

The blood flow comparison of color ultrasound images before and after use of motherwort injection is shown in Figure 5.

After one week of treatment, vaginal bleeding was significantly less than that in the control group.

The results of comparison of vaginal bleeding time and uterine hemorrhage between the two groups of patients given in Table 2 provide that after 1 week of treatment, the vaginal bleeding time of the observation group was significantly shorter than that of the control group, the number of cases of uterine hemorrhage was significantly reduced compared with the control group, and the difference was statistically significant (*P* < 0.01).

Comparison of clinical efficacy between the two groups of patients given in Table 3 provides that after 1 week of treatment, the cure rate and total effective rate of the observation group were 64.98% and 97.95%, respectively, and the control group was 30.08% and 80.14%, respectively. The cure rate, total effective rate, and overall curative effect of the observation group were better than those of the control group, and the differences were statistically significant (*P* < 0.01).

## 5. Conclusion

In this study, after the treatment group was treated with oxytocin combined with motherwort granules after drug abortion, vaginal bleeding time and bleeding volume were significantly lower than those of the control group (*P* > 0.05); ultrasound images clearly show that the amount of bleeding is reduced; it is suggested that oxytocin combined with motherwort can effectively reduce the postmedical abortion, vaginal bleeding time, and bleeding volume, conducive to postoperative recovery. Motherwort has a significant effect on postoperative vaginal bleeding and can significantly shorten the time of vaginal bleeding and reduce the occurrence of complications such as uterine hemorrhage and infection, which is conducive to the recovery of patients; at the same time, it helps to improve the quality of life of patients and is worthy of clinical application.

## Figures and Tables

**Figure 1:** The main causes of maternal death in my country.

**Figure 2:** High-risk factors leading to uterine weakness.

**Figure 3:** The incidence of bleeding in different delivery methods.

**Figure 4:** Comparison of motherwort injection (a) before use and (b) after use.

**Figure 5:** Color ultrasound images of *Leonurus* injection (a) before and (b) after use of motherwort injection.

**Table 1:** The difference between *Leonurus* injection and oxytocin.

	Motherwort injection	Oxytocin
Site of action	Total uterine contraction	Lower contraction is weaker
Action time	2–5 min, half-life 6 h	Rapid onset, with a half-life of 5 min

**Table 2:** Comparison of vaginal bleeding time and uterine hemorrhage in the two groups.

	*N*	t_Vaginal bleeding_/d	*n*_Uterine hematocele_ (*p*/%)
Control group	60	10.25 ± 0.1	15
Observation group	60	7.36 ± 0.1	3

**Table 3:** Comparison of clinical efficacy of patients in groups.

	*N*	Cure	Efficient	Invalid	Always effective
Control group	60	21	30	10	51
Observation group	60	42	17	1	59

## Data Availability

The data used to support the findings of this study are available from the corresponding author upon request.
